# Research on the Impact of Livelihood Capital by the Honghu Fishermen's Willingness to Quit Fishing

**DOI:** 10.1155/2022/1900301

**Published:** 2022-10-03

**Authors:** Yu Zhou, Zhaohua Li, Liya Zhao

**Affiliations:** Faculty of Resources and Environmental Science, Hubei University, Wuhan 430062, China

## Abstract

Aiming at the livelihood of fishermen under the fishing prohibition policy, quantitative research methods were used to explore the relationship between the willingness to quit fishing and livelihood capital. With reference to 609 survey data from 20 fishing grounds in 2 counties and cities of Hubei Province, this paper explores the necessity of convincing fishermen in the Yangtze River to quit fishing and evaluates the impact of livelihood mode on Honghu fishermen's willingness to quit fishing by means of structural equation model based on the sustainable livelihood framework developed by the UK Department for International Development. The results showed the following conclusions: (1) The proportion of fishermen who are willing to participate in quitting fishing is 66.7%, indicating that fishery production is still the main source of livelihood for many fishermen. The overall willingness of fishermen to quit fishing is strong, and fishermen have realized the importance of protecting fishery resources. (2) There is a strong correlation between the indicators of livelihood capital and the willingness of fishermen to quit fishing. Among them, the human capital has the most significant impact on fishermen's willingness to quit fishing for some compensation from public power. The research conclusion is helpful for the government to improve the fishing prohibition policy in a targeted manner and mobilize the enthusiasm of fishermen to protect fishery resources.

## 1. Introduction

The Yangtze River is the third largest river in the world and the largest river in Asia. It has wealthy aquatic biological resources and is a treasure house of precious freshwater organisms on the Earth. According to statistics, the Yangtze River in China has a total length of more than 6,300 kilometers and a basin area of 1.8 million square kilometers. There are more than 4,300 aquatic organisms distributed in the Yangtze River Basin, of which 424 species (subspecies) are fish, accounting for about 29% of the 1,450 species of freshwater fish in China. The Yangtze River also has many rare and unique species of fish. Among them, 11 species are under national key protection and more than 170 species are unique [1]. Therefore, the responsibility of protecting the fishery resources of the Yangtze River is particularly important.

In recent years, with the development of society and economy, the Yangtze River Basin has established new water conservancy facilities, reclaimed lakes and reclaimed land, and overfishing, which has greatly reduced the output and quality of fishery resources. According to statistics from the State Fisheries Administration, the number of seedlings of the main economic fishes in the Yangtze River has dropped from 30 billion to 200 million, and “fish-free zones” have even appeared in many river basins. Fishery catch has fallen from more than 400,000 tons per year in the 1950s to less than 100,000 tons per year the specific year the estimate of 100,000 tons was made. The number of endangered fish species listed in the *China Red Data Book of Endangered Animals* has reached 92 species. Moreover, the species listed in the appendix of the *Convention on International Trade in Endangered Wild Fauna and Plants* approached 300 species [2].

Honghu Lake is the seventh largest freshwater lake in China with an area of 355 square kilometers (Figure 1). As an important lake in the middle reaches of the Yangtze River, Honghu lake is the habitat of many waterfowls and has plentiful fishery resources. Before the 1960s, Honghu Lake was connected to the Yangtze River. The water of the lake fluctuated with the river water. There were 114 species of freshwater fishes, including Chinese sturgeon, white sturgeon, and brown fish. After the 1960s, due to overfishing by fishermen, the fishery resources of Honghu Lake were greatly reduced. There are 57 species of freshwater fishes, and carps accounted for 58.5% [3]. Among these fish resources, piscivorous fish accounted for 57.4%, such as yellow catfish, rice field eel, and herring. Omnivorous fish accounted for 22.2%, such as crucian carp, snakehead, and loach. Only 7.4% fed on aquatic plants, such as the grass carp and bream. There were 7 species of mackerel and carp that fed on algae and decay [4]. Also, only two kinds of silver carp and bighead carp eat plankton. Data illustrate the types of fish resources in Honghu Lake have been decreasing in recent years. Moreover, next to half of the fish populations are on the verge of extinction. The changes in the quantity and species composition of fish resources directly affect the livelihood capital of fishermen and have an impact on the production and life of fishermen.

There are 164,000 fishermen in the entire Yangtze River basin. The Yangtze River flows through more than ten provinces, of which Hubei is the longest. Moreover, Honghu is the place with the most traditional fishermen in Hubei Province. To this end, the state has successively issued a series of policies to strengthen the protection of fishery resources in the Honghu Lake Basin. In 2019, the Honghu Government issued a work plan for the compensation for fishermen quitting fishing, which detailed the compensation standards for quitting fishing in Honghu. For fishermen whose fishing rights are confiscated, compensation of 40,000 yuan per boat will be given. For fishermen whose fishing boats and fishing gear have been expropriated, and switch to other industries, the compensation for changing production will be 5,000 yuan per boat. After the fishermen quit fishing, they can enjoy a 19-month transitional living allowance of 1,000 yuan per boat per month.

Since the implementation of the fishing prohibition policy, 13,000 fishing fishermen in Honghu Lake have quitted fishing and 16,000 fishing boats have quitted fishing. These fishermen are facing survival difficulties [5]. The challenge of how to deal with the livelihood of fishermen who have been affected has become an important issue, which needs to be studied and resolved.

## 2. Literature Review

There have been rich accumulations of research on livelihood capital, but there are few research studies on fishermen's livelihood methods. Livelihood capital refers to the available resources that can be reserved, interchanged, or allocated for people's survival to generate income streams or benefits [6]. In the sustainable livelihood analysis framework of the UK Department for International Development (DFID), livelihood capital includes five types: natural capital, physical capital, financial capital, human capital, and social capital [7]. The most relevant aspects of this research are the sustainable livelihoods of farmers and herders. These studies provide a good reference for this paper.

As the main providers of ecosystem services, farmers' livelihood capital affects the use of natural resources and plays a vital role in the implementation of environmental protection policies. To this end, many scholars have carried out research on farmers' willingness to protect the ecological environment from aspects of livelihood, ecological perception, and information transmission [8, 9]. On the one hand, it has become the consensus of the academic community to take targeted ecological protection measures based on the farmers' livelihood status, willingness to receive compensation, and ecological perception [10, 11]. Among them, developing countries have conducted extensive research studies on farmers' livelihood capital [4]. For example, de Sherbinin et al. compared the difference in livelihood conditions between the Amazon region and the sub-Saharan region [12]. However, some scholars have found through the study of farmers' livelihood capital that maintaining the original quality life of farmers plays an important role in the implementation of ecological compensation policies. On the other hand, the family livelihood capital of farmers is an important guarantee for their survival. Only when long-term livelihoods are guaranteed, can farmers have extra energy to pay attention to changes in the ecological environment and further generate a willingness to protect [13]. Therefore, it is particularly important to identify the livelihood capital available to farmers and to deeply study the relationship between the livelihood capital of farmers' families and the willingness to participate.

Fishermen who have quitted fishing are one aspect of labor transfer research in the field of fisheries. In the study of population migration, Stark and Bloom emphasized the role of individuals value choices in migration willingness, but he transferred the subject of migration from rural labor individuals to rural families [14]. Because individual choice is actually the result of family division of labor and decision-making and distribution. Rural labor migration is more often a decision made based on the overall consideration of the family [15, 16]. From this, Stark concluded the new economic migration theory. The core value of the New Economic Migration Theory lies in positioning the main body of migration decision-making in the family and then adjusting the migration decision-making variable from income level to income stability. This means that under weaker institutional constraints, migration may be inevitable, because the risk of employment income in the nonagricultural sector is significantly lower [17, 18]. The theory of new economic migration has a guiding role in the relationship between fishermen's livelihood capital and the willingness to quit fishing.

Fishermen who have quitted fishing are related to many factors. In terms of theoretical research, Akerlof and Kranton explored how identity affects personal interactions through a simple game-theoretic model. In this model, the economics of sexism in the workplace, poverty and social exclusion, and the division of labor at home are incorporated [19]. Capital is a factor that cannot be ignored. Based on a survey of more than 1,400 fishing vessel owners on the U.S. West Coast, Holland et al. noted that the nonmonetary and monetary aspects of fishing are related to job satisfaction, fisherman status and social capital, and participation in fishing have a clear impact. Nonmonetary job satisfaction, social capital, and status were correlated with willingness to give up higher incomes to become fishermen [20]. Hanna and Smith conducted a survey of captains of a trawler and found that the fishermen were the same in their motivations and decisions. They are lacking of foresights and ignore the impact of their fishing on fishery resources. The potential cost of providing false information to fishermen in fishery resource utilization patterns [21]. Plagányi et al.pointed out that in the field of fisheries, most research has focused on industry, ignoring the contribution of small and local hunters and fishermen to global resource use. For many indigenous groups, it is local autonomy, not capitalism, that influences the views and aspirations of fishermen. In capitalist countries, market-based management plans may get higher scores. However, in a country that places high value on public ethics, it can adversely affect the coherence and fairness of society [22].

Quitting fishing willingness are also related to the fisherman's financial status and personal characteristics. Cinner and McClanahan investigated the willingness of Kenyan fishermen to stop fishing and the impact of socioeconomic conditions assuming a decline in catches and found that fishermen from poor households were less likely to experience a severe decline in fisheries. Withdrawal from fisheries is consistent with the literature on poverty traps showing that poor people are unable to mobilize the necessary resources to overcome shocks or to overcome chronic low incomes. The findings of this study confirm that targeting the poorest fishermen to create wealth and jobs can help reduce fishing efforts in overfishing industries. However, in order to do this, it is necessary to have an understanding of the socioeconomic environment in which the fisherman operates [23]. Pollnac and Poggie surveyed commercial fishermen, charterers, and fish factory workers for job satisfaction, correlations between fishing type, crew size, etc., and their personal characteristics [24]. Smith employed a cognitive approach to distinguish the characteristics and relative satisfaction rewards of commercial and recreational salmon fishermen. This research suggests that a fishing-like experience is critical for some commercial salmon fishers. For some commercial fishermen, this pleasant element brings a special kind of thrill. The research aims to explore how to best optimize the allocation of labour and capital and limit work in fisheries across different operations [25].

The formulation of the fishing prohibition policy has economic considerations and it is a game between the government, fishermen and the ecological environment. Anderson explored the logic of fisheries WSB and its implications for policy. A detailed model shows how the surpluses across sectors are linked and how they change across output levels [26]. Durrenberger reviewed the challenges of the Schaefer-Gordon fishery management model to biological assumptions and pointed out that its economic assumptions also have loopholes. Combining data from other fisheries and Mississippi river crab with comparative data, according to the method proposed by Chayanov, show that Chayanov's model is characteristic of Mississippi shrimpers [27]. Smith and Hanna proposed two approaches to fisheries research, community research, and occupational focus. Occupational analysis shows how fishing differs from other activities, as well as the differences between fishing activities. The study shows that within a fishery, community factors differentiate the behavior of fishermen. The reason why the community factor persists lies in the pattern of information transfer. The community is more characterized by face-to-face interaction, which is conducive to the transmission of ideas. The study focused on trawlers in Oregon [28].

Previous research results on the influencing factors of willingness and farmers' livelihoods are abundant, but there are few discussions and studies on fishermen's livelihoods and willingness to quit fishing. Throughout these literature studies, the selected influencing factors can be divided into individual characteristics, family characteristics, production characteristics, and cognitive characteristics. Pang and Jin constructed an equivalent function of fishermen's willingness to pay compensation for fishing prohibition and analyzed the influencing factors of fishermen's willingness to pay by binary logistic regression model. The study concluded that through the parameter estimation of the equivalent utility function, incorporating objective conditions into the estimation category can restrain the subjective assumptions of the interviewed fishermen to a certain extent, thereby making the estimation results closer to the objective facts. Fishermen's willingness to pay is affected by individual characteristics, family characteristics, production characteristics, and subjective cognition [29]. Chen and Liu based on the survey data and used the binomial distribution logistic regression model to analyze the willingness of fishermen to quit fishing production activities and their influencing factors in the middle and lower reaches of the Yangtze River. The willingness of fishing activities in the Yangtze River fishery has a positive impact; the number of households and fishing income have a negative impact on the willingness of fishermen to quit fishing in the Yangtze River fishery [30]. In terms of fishermen's livelihood, some scholars have studied the willingness of fishermen to quit fishing by referring to the research results of sustainable livelihood and farmers' livelihood. Lei et al. conducted a field investigation on fishermen's willingness to quit fishing and sustainable livelihood capital in the Poyang Lake area and used a binary logistic regression model to analyze the results. It is concluded that the natural capital and financial capital have a significant negative impact on the willingness to withdraw from arrest [31].

The research content of this paper includes the following: (1) explaining the related concepts of the research, sorting out the theoretical basis, and putting forward research hypotheses. (2) Conducting field surveys of Honghu fishermen, the main content includes the content design of the questionnaire survey, the actual content and scope of the survey. (3) Based on the survey samples of fishermen's willingness to accept, relying on the sustainable livelihood framework theory and using structural equation models to analyze the relationship between fishermen's livelihood capital and willingness to quit fishing to provide suggestions for the government to formulate corresponding fishing prohibition policies.

## 3. Research Hypothesis and Variables

### 3.1. Research Hypotheses

Livelihood capital refers to a way of life realized or maintained by farmers' earning ability, assets, and income activities. The sustainable livelihood framework theory developed by the UK Department for International Development includes five aspects, natural capital, physical capital, financial capital, human capital, and social capital [32, 33]. This framework emphasizes the persistence of human-centeredness, with vulnerability as the research background. Farmers' livelihood capital will have an impact on the choice of their livelihood strategies due to changes in some external factors. The core lies in the relationship between livelihood capital and livelihood strategies.

Fishermen's livelihood capital can bring benefits to fishermen's production activities and social activities to ensure their subsequent livelihood value. The natural capital refers to the natural resources such as cultivated land, ponds, and forest land owned by farmers' families. For fishers, natural capital refers to waters, wetlands, and other natural resources and environmental services that create value for fishermen's survival in a certain period of time. Financial capital refers to the liquid assets accumulated by fishermen to maintain their livelihoods. Physical capital refers to the production equipment (fishing boats and the fishing gear) and living infrastructure needed by fishermen in fishing activities. Human capital refers to the quantity and quality of fishermen's labor in production activities [34]. Social capital refers to the social resources and network that can be used by fishermen in their livelihood activities [35]. These capitals are interrelated and they interact with one another under the action of external force and internal self and become the decisive factor for fishermen to quit fishing. As far as the fishing prohibition policy is concerned, fishermen's family livelihood is their livelihood strategy and a vital basis for realizing their livelihood goals. The choice of fishermen's livelihood behavior and its result are composed of system, policy, and capital, wherein the livelihood capital status of fishermen's families plays a decisive role in the choice of fishermen's livelihood behaviors. It directly affects the fishermen's willingness to quit fishing and then affects the fishing-withdrawal behavior [36]. On the strength of the structural equation model, fishermen's livelihood mode is included in the measurement index of willingness to quit fishing, so that study the impact of livelihood capital on the willingness to quit fishing. The theoretical framework analysis chart is shown in Figure 2.

**Hypothesis 1 .**

The better the natural capital endowment of fishermen's families is, the lower their willingness to quit fishing. Generally, natural capital is the expression of fishermen's agricultural and natural resources endowment, chiefly including land, waters, fishery resources, and other natural resources. Following the decline of fishery resources in the basin, fishermen's livelihood method is pursuing seine farming. Families have less cultivated land and are not good at farming. The higher their natural capital endowment is, the more economic benefits are expected to be acquired by livelihood methods acquired by livelihood methods associated with fishing, and the lower their willingness to quit fishing is.

**Hypothesis 2 .**

The higher the physical capital level of fishermen's families is, the lower their willingness to quit fishing. The higher the physical capital level of the vast majority of fishermen's families, the more willing to choose a fishery-based livelihood model, the stronger the dependence on fishery. Therefore, fishermen are more reluctant to give up fishery under the high level of material capital.

**Hypothesis 3 .**

The better the financial capital of fishermen's families is, the stronger their willingness to quit fishing. Financial capital includes two forms: one is financial capital, such as bank loans, savings, and other financial derivatives; the other is noninterest-bearing financial capital [37], such as fishermen's income, government subsidies, etc. The more profitable financial capital a fisherman has, the less pressure his life will be, and the more time and energy he will have to focus on things other than his livelihood.

**Hypothesis 4 .**

The more abundant the human capital of fishermen's families is, the stronger their willingness to quit fishing. In the 1960s, American scholar Schultz believed that human capital is a kind of capital embodied in people that can bring income to the future [38]. In the framework of sustainable livelihoods, human capital is determined by factors such as the number of family laborers, knowledge, skills, and health status. The human capital of fishermen determines the ability of fishermen to master nature, material, finance, and social capital, and is the basis of the other four types of capital. The better the farmers' social capital is, the more they realize the significance and severity of the fishing prohibition policy and protecting fishery resources. Thus, the better the social capital of fishermen's families is, the stronger their willingness to quit fishing and change jobs.

**Hypothesis 5 .**

The better the social capital of fishermen's families is, the stronger their willingness to quit fishing. Bourdieu proposed that social capital is a complex of realized or potential resources, and resources are related to the group membership [39]. Social capital is a kind of social relationship, which manifests in the new people, social relationships and rules established between people based on the blood relationship, geographical relationship and emotional relationship. Social capital is a bridge between fishermen and the outside world, and is a product of the external environment. See Table 1.

### 3.2. Variable Selection

Through the theoretical analysis, drawing lessons from the results of variable selection and scale design of the related studies, and in consideration of the actual situation of investigation, 17 topics are designed to measure fishermen's “willingness to quit fishing” and “livelihood capital,” in which livelihood capital is chiefly composed of five parts: natural capital, physical capital, financial capital, human capital and social capital, and the meanings and assignment of variables are presented in Table 2. Fishermen's willingness to quit fishing is a binary dependent variable that takes a value of one if the fishermen expressed a willingness to quit fishing and a value of zero otherwise.

## 4. Model Building and Data Sources

### 4.1. Model Building

The greatest superiority of structural equation model is that it can deal with multiple dependent variables simultaneously. A key advantage of structural equation modeling it that allows for simultaneous estimation of latent variables and their relationship to a dependent variable of interest and allows for measurement error in the latent variables [40]. Thus, it is more suitable for simultaneous analysis of multi-cause and multiresult problems with the structural equation model. The SEM constructed in this thesis is as follows:

(1) $$\begin{array}{c} \eta =\alpha \eta +\delta \xi +\gamma . \end{array}$$

Equation (1) is a structural equation used to define the linear correlation between latent independent variables and endogenous latent variables; *η* is an endogenous latent variable, meaning fishermen's willingness to quit fishing; *α* is the relationship between endogenous latent variables; *δ* is the impact of exogenous latent variables on endogenous latent variables; *ξ* is exogenous latent variable, which refers to the livelihood capital of fishermen's families; *γ* is the error term of endogenous latent variable.

(2) $$\begin{array}{c} Y=\wedge {}_{y}\eta +\varepsilon , \end{array}$$

(3) $$\begin{array}{c} X=\wedge {}_{x}\xi +\beta . \end{array}$$

Equations (2) and (3) are measurement models, which are used to embody the relationship between endogenous latent variables and observable variables. *Y* is the objective index of endogenous latent variables, that is, the index of fishermen's willingness to quit fishing; ∧*y* is the factor load between endogenous latent variables and observed variables; *X* is the observable variable of exogenous latent variable, that is, the index reflecting livelihood capital; ∧*x* is the factor load between exogenous latent variable and observed variable, and *β* means the measurement error of each observed variable of exogenous latent variable [39].

Logistic regression model is often used in data mining, automatic disease diagnosis, economic forecasting, and other fields. According to the different types of dependent variables, logistic regression analysis is divided into binary regression analysis and multiple regression analysis. According to the needs of this study, the fishermen's willingness to quit fishing has only two situations: willingness and unwillingness. So, the binary logistic regression model is more suitable.

Let *Y* be the dependent variable. When *Y* = 1, it means that the fishermen are willing to quit fishing; when *Y* = 0, it means that the fishermen are unwilling to quit fishing. The five livelihood capitals that affect *Y* are used as independent variables, namely, social capital (*X*1), human capital (*X*2), financial capital (*X*3), physical capital (*X*4), and natural capital (*X*5).

### 4.2. Samples and Data

Honghu Lake is located in the middle reaches of the Yangtze River and is the largest lake in Hubei Province. The program to incentivize fishermen to quit fishing in the Yangtze River Basin involves 79 traditional fishing villages in Honghu, with more than 100,000 fishermen. There are 22,000 fishing boats in Hubei Province, including 16,000 fishing boats in the two counties along the Honghu Lake, accounting for 71% of the total number of fishing boats [1]. The research team visited 20 key fishing grounds along the lake in the Honghu Basin: 6 townships including Chahe Town, Qujiawan Town, Luoshan Town, Xindi Street, Binhe Street, and Shakou Town in Honghu City, with a total of 15 fishing grounds. There are 3 townships in Jianli County, Qiaoshi Town, Bianhe Town, and Qipan Township, with a total of 5 fishing grounds. According to the statistics of the local fishery administration, all fishing boats in Honghu City account for more than 70% of the fishing boats in the entire lake. In response to the special circumstances of fishermen, we choose participatory rural assessment (PRA) tools such as questionnaire surveys, observation methods, and small seminars to help fishermen understand the questions more accurately, thereby increasing the response rate of the questionnaire. At the same time, it can also strengthen fishermen's understanding of the policy and play a role in promoting the policy.

The data used herein come from the household survey conducted in Honghu City and Jianli City of Jingzhou City from August 30 to October 10, 2020. The sample fishing grounds were determined by a random sampling method, and the researcher and fishermen were interviewed face to face. A total of 639 questionnaires were distributed and 609 valid questionnaires were acquired, with an effective rate of 95.31%, including 496 questionnaires in Honghu City and 113 in Jianli City (Table 3).

Among the 609 Honghu fishermen survey samples, 406 have expressed their willingness to quit fishing, accounting for 66.7% of the total sample. 203 households were unwilling to quit fishing, accounting for 33.3% of the total sample. It can be seen that the vast majority of Honghu fishermen are willing to quit fishing activities for some form of compensation.

Compensation for quitting fishing refers to the compensation of public power to fishermen who quit the Honghu Lake for fishing and breeding. According to the survey, the compensation for quitting fishing consists of housing subsidies, compensation for scrapped fishing boats, and compensation for the removal of the aquaculture purse seine in the Honghu Lake area. The housing compensation is 70,000 yuan per household and 20,000 yuan or 10,000 yuan per person (20,000 yuan for urban houses and 10,000 for rural houses). Fishing boat compensation means that the fishing boat is redeemed according to market valuation and the boat is confiscated. The demolition of the lake area will be compensated by 11050 yuan/household.

The statistical analysis of the samples suggests (Table 4) that those who chiefly live on fishing are men, making up 82.8%, whose ages are principally concentrated in 41–60, accounting for 51%. Their education level is mostly junior high school and below, occupying 82.3%; the family population is 5-6 people, up to 41.5%. The net income from family business is 81109.65 yuan, the per capital annual income is 17000 yuan, and the per capita farming area is 12,000 m^2^. The fishermen interviewed are characterized by male labor force, aging population structure and low average education level. Meanwhile, the average income of the interviewed fishermen's families is comparatively high. And the aquaculture area is large, which reveals that the fishing investment and income are high.

## 5. Results and Analysis

### 5.1. Reliability Analysis and Validity Test

Reliability reveals the reliability of measurement, and it chiefly embodies the true degree of the measured data based on the consistency or stability of the results acquired by the test tools [41]. In this thesis, SPSS24 software is applied to test the internal consistency of 17 observed variables in the questionnaire. The reliability test index Cronbach's alpha coefficient is 0.87. Cronbach's alpha coefficients of each latent variable are all greater than 0.7. The total reliability coefficient Cronbach's alpha value of the scale is up to 0.926, which means that the reliability of sample data acquired by the questionnaire is pretty good.

In a bid to further test whether the overall internal structure of the questionnaire is reasonable, this thesis analyzes the exploratory factors of the latent variables. In the measurement model, the standard factor load coefficients of all latent variables and observed variables are greater than the threshold value of 0.5. The path coefficients of the selected measurable variables and latent variables are significant at the level of 1%, revealing that the internal consistency of each variable is relatively good. Meanwhile, the validity test suggests that KOM (Kaiser-Meyer-Olkin) value is 0.847; when it is greater than 0.6, the approximate Chi-square value of Bartlett spherical test is 1861.901, the degree of freedom is 465. It is significant at the statistical level of 1%, demonstrating that the structural validity of the questionnaire is relatively good and it is suitable for factor analysis. A total of 6 common factors were selected from 17 topics, and the cumulative variance variation is 73.105%, which is relatively ideal for explaining the original data. Apart from that, the composition reliability CR is between 0.711 and 0.87, which is higher than the threshold of 0.7. According to Table 5, The average variance extraction AVE is between 0.519 and 0.603. The questionnaire is provided with convergence validity.

### 5.2. Test of the Overall Fitness of the Model

The fitting degree of the model serves as the vital basis for testing whether the theoretical model is scientific or not [42] There is a certain scope of application for TPB theory. While the sample data are in line with the requirements of model construction, this thesis fits the structural equation model with AMOS25.0 software. As indicated by the test indexes of the overall fitness of the model, the values of each index in the absolute fitting index and the relative fitting index of the model are within the suggested range of values, which presents that the overall fitness of the model is fairly good [43] according to Table 6.

### 5.3. Results and Discussion

The standardized path map of the impact of livelihood on fishermen's willingness to quit fishing is acquired by virtue of the research model and AMOS25.0 software. As shown in Table 7, the path coefficients of all latent variables in the model have passed the test of 1% significance level, which reveals that fishermen's family livelihood exerts a significant impact on their willingness to quit fishing, and the above hypotheses have been confirmed. Specific analysis is as given below:

1. The total path coefficient of natural capital to fishermen's willingness to quit fishing is −0.581 as shown in Table 7. It has passed the test of 1% significance level, suggesting that the more abundant natural capital is, the lower the fishermen's willingness to quit fishing. That is, H1 is tested to be valid. In light of the estimation results of the standardized path coefficient, the culture area of paddy fields contracted by the fishermen contributes the most to natural capital (standardized coefficient is 0.792), followed by the culture area of net cages (standardized coefficient is 0.756) and cultivated land area (standardized coefficient is 0.682). Both the aquaculture area and the catch will inhibit the willingness of fishermen to quit fishing. Among the 609 fishermen's households surveyed, the fishermen use Honghu Lake as a production site and the area of arable land is relatively small. The carrying capacity of lake resources is determined by the aquaculture area and the number of fish caught. The larger the aquaculture area owned by fishermen, the stronger the carrying capacity of the lake, the lower the risk of overloading, and the less likely fishermen to quit fishing. Affected by climate and policies, the annual catch of fishermen will change, and when the catch is greater, the willingness of fishermen to quit fishing will be lower [35].
2. Table 7 shows that the total path coefficient of physical capital to fishermen's willingness to quit fishing is −0.498, which has passed the test of 1% significance level. The results reveal that the more abundant the physical capital of fishermen, the lower their willingness to quit fishing. That is, H2 is tested to be valid. Viewing from the estimation results of standardized path coefficient, the distance between fishermen's homes and Honghu Lake contributes the most (standardized coefficient is 0.861), followed by the number of special equipment (standardized coefficient is 0.84) and finally the housing conditions (standardized coefficient is 0.825). It may be mainly because the physical capital of fishermen's families is mainly based on the value of fishing boats, fishing gear and houses. When they have more special fishing equipment, their willingness to quit fishing will be lower.
3. As shown in Table 7, the total path coefficient of financial capital to fishermen's willingness to quit fishing is −0.362, which has passed the test of 1% significance level. It indicates that the more financial capital of fishermen, the stronger their willingness to quit fishing and changing jobs. That is, H3 is tested to be verified. Financial capital can reflect the economic strength of a fisherman's family. When the financial capital of a fisherman's family is more significant, its dependence on fishing becomes weaker, and the willingness to participate in quitting fishing is strong.
4. Inspired by the estimation results of standardized path coefficient, free cash assistance opportunities (standardized coefficient is 0.861) bring more contribution than the annual income of fishermen's families (standardized coefficient is 0.646) and the difficulty of gaining loans (standardized coefficient is 0.623). The higher the family cash income of fishermen, the stronger the willingness to quit fishing. The reasons may be: household income is the indicator that best reflects the livelihood of fishermen. The higher the cash income, the wealthier the family. Although quitting fishing will reduce the income of fishermen, fishermen with high family income are more able to bear the loss of income caused by quitting fishing to protect water ecological resources. And the marginal effect of quitting fishing on the income loss caused by it is relatively small, but the higher the family income, the higher the pursuit of the quality of life and the environment of the fishermen, and they are often more willing to improve the lake ecological environment [35].
5. According to Table 7, the total path coefficient of human capital to fishermen's willingness to quit fishing is −0.592, which has passed the test of 1% significance level. In comparison with natural capital, physical capital, financial capital and social capital, human capital exerts the most distinct impact on fishermen's willingness to quit fishing, which demonstrates that the more human capital the fishermen's families possess, the stronger their willingness to quit fishing and changing jobs, that is, H4 is tested to be verified.
6. In light of the estimation results of standardized path coefficient, the educational level of the main family labor force (standardized coefficient is 0.899) contributes the most to human capital, followed by the number of family population (standardized coefficient is 0.83), and finally the proportion of labor force in the family population (standardized coefficient is 0.712). For fishermen, the larger the family population, the more surplus labor outside the fishery. Therefore, the larger the proportion of other income of the whole family, the higher the dependence on nonfishery employment. At the same time, under the dual pressure of the deteriorating lake ecology and the relatively low efficiency of fisheries, the labor-rich fishermen's families reduce their dependence on fisheries through quitting fishing. It is more likely to liberate labor from fishery production.
7. The total path coefficient of social capital to fishermen's willingness to quit fishing is 0.41, which has passed the test of 1% significance level according to Table 7. It's suggesting that the more social capital the fishermen own, the higher their willingness to quit fishing. That is, H5 is tested to be valid. Good social relations and abundant information resources make fishermen more fully aware of the fishing prohibition policy, and the greater the willingness to participate in quitting fishing.

Suggested by the estimation results of standardized path coefficient (Figure 3), the biggest contribution to human capital is conditioned by whether there are village cadres among family members (standardized coefficient is 0.899s), followed by whether there are township cadres among relatives (standardized coefficient is 0.830), and finally the proportion of labor force in the family population (standardized coefficient is 0.712). The reason may be that the more social capital is accumulated, the more resources of fishermen's social relations, the more channels they have to receive information, and the more abundant the social communication relations they are in. Good social relations and abundant information resources enable fishermen to be more fully aware of the fishing prohibition policy, and the stronger their willingness to quit fishing will be.

Further, a binary logistic regression model was used to analyze the relationship between fishermen's willingness to quit fishing and livelihood capital, and the results are shown in Table 8.

Table 8 shows that the Sig values of the five types of livelihood capital are all less than 0.05, indicating that each type of livelihood capital is closely related to the willingness of fishermen to quit fishing. Among them, the correlation coefficients of natural capital, physical capital, and social capital are positive (0.841, 1.216, 1.395), indicating a positive correlation with fishermen's willingness to quit fishing. The correlation coefficients of human capital and financial capital are negative (−0.663, −1.251), indicating a negative correlation with the willingness of fishermen to quit fishing. The social capital result is consistent with that of the structural equation model. Moreover, it is consistent with the research results of Holland et al. [20], as well as the research result of Plagányi et al. [22], the willingness of fishermen to quit fishing is closely related to capital factor. Lei et al. [31] and Pang and Jin [29] both discuss similar issues, but the study area and estimation method are different from this study, as shown in Table 9.

## 6. Conclusion

Fishery resources are an effective starting point for the restoration and protection of the Honghu Lake's water ecology. By motivating fishermen to quit fishing, it is an inevitable choice to manage the ecological environment of the Yangtze River Basin. Based on the theory of planned behavior, this paper uses the survey data of 609 fishermen in Honghu Lake to study the influence of natural capital, physical capital, financial capital, human capital, and social capital on the willingness of quitting fishing from the perspective of livelihood methods. The main conclusions of the research are as follows:

First, from the overall sample statistics, 66.7% of fishermen expressed their willingness to participate in quitting fishing, while only 33.3% of fishermen expressed their unwillingness. This also shows that as a traditional fishery province in Hubei Province, fishery production is still the main source of livelihood for many fishermen. The overall willingness of fishermen to quit fishing is relatively strong, and fishermen realize the importance of protecting fishery resources.

Second, there is a strong correlation between the indicators of livelihood capital and the willingness of fishermen to quit fishing. Among them, human capital has the most significant impact on fishermen's willingness to participate in quitting fishing. This significant effect is the same as the research results of Liu and Yu [35] and Pang and Jin [29]. It is unanimously agreed that the education level of family labor produces a significant impact on fishermen's willingness to quit fishing.

The above mentioned conclusions suggest that the government should consider the current display of fishermen's livelihood differentiation, as well as the impact of fishermen's livelihood changes on the willingness to quit fishing, and improve the fishing prohibition policy in a targeted manner, so as to mobilize the enthusiasm of fishermen for farmland protection. In order to ensure the smooth implementation of the Honghu fishing prohibition policy, the publicity of the fishing prohibition policy should be strengthened to let more fishermen understand the purpose of the fishing prohibition policy and further improve the fishermen's level of awareness. The human capital of fishermen is a key factor in motivating fishermen to participate in quitting fishing. Among them, the positive impact of fishermen's diversification of livelihoods is the most significant. Therefore, the government should focus on guiding the cultivation of ecological industry development and strengthen fishermen's livelihood skills training to reduce fishermen's influence on fishery. The degree of dependence on resources fundamentally solves the problem of fishermen's long-term livelihoods, thereby realizing the sustainable development of fishery resources.

## Figures and Tables

**Figure 1:** Study area. Data resource: Hubei provincial department of natural resources.

**Figure 2:** Theoretical framework analysis chart. Data resource: processed from survey.

**Figure 3:** Structural equation model and diagram of standardized path coefficient. Data resource: processed from survey; “*∗*,” “*∗∗*”, and “*∗∗∗*” represent the significance levels of 0.1, 0.05, and 0.01, respectively.

**Table 1:** Hypothesis on observed variables.

Hypothesis	Latent variable	Correlational relationship
H1	Natural capital ⟶ Fishermen's willingness to quit fishing	Negative correlation
H2	Physical capital ⟶ Fishermen's willingness to quit fishing	Negative correlation
H3	Financial capital ⟶ Fishermen's willingness to quit fishing	Positive correlation
H4	Human capital ⟶ Fishermen's willingness to quit fishing	Positive correlation
H5	Social capital ⟶ Fishermen's willingness to quit fishing	Positive correlation

Data resource: processed from survey.

**Table 2:** Index system and assignment of fishermen's livelihood capital.

Livelihood capital	Measured variable	Meaning and description of assignment
Natural capital	Culture area of paddy field	Breeding area of actual paddy fields of families
	Cultivated area	Actual cultivated land area per capita
	Fishery input-output ratio	Fishing input/fishing output

Physical capital	Housing type and area	Concrete house = 1.0, brick-wood house = 0.75, civil house = 0.5, shed circle = 0.25; 5 rooms and above = 1.0, 4 rooms = 0.75, 3 rooms = 0.5, 2 rooms = 0.25, 1 room = 0
	Number of fishing boats	Wooden boat = 1, mixed structure boat = 2, steel boat = 3, glass fiber reinforced plastic boat = 4, aluminum alloy boat = 5, steel mesh cement boat = 6
Financial capital	Annual income of fishermen's families	RMB 90,000 or more = 6; RMB 70,000–90,000 = 5; RMB 50,000–70,000 = 4; RMB 30,000–50,000 = 3; RMB 10,000–30,000 = 2; less than RMB 10,000 = 1
	Opportunity to get a loan	Very difficult = 1, relatively difficult = 2, general = 3, relatively easy = 4, easy = 5
	Opportunities for unpaid cash assistance	Yes = 1, no = 0

Human capital	Proportion of labor force to family population	Proportion of number of labor force to the total number of families
	Educational level of the main labor force in the family	Illiteracy = 1, primary school = 2, junior high school = 3, senior high school or technical secondary school = 4, junior college or above = 5
	Non-agricultural employment skills of householder	Yes = 1, no = 0

Social capital	Number of relatives and friends	Number of relatives and friends around Honghu
	Level of trust in people around the fishery	Very trust = 1, relatively trust = 0.75, general = 0.5, not very trust = 0.25, very distrust = 0
	Degree of understanding of the fishing prohibition policy	Very unknown = 1, unknown = 2, general = 3, known = 4, very well-known = 5

Data resource: processed from survey.

**Table 3:** Distribution of survey samples.

Area	Fishery name	Total *N*.	Valid *N*.	Effective ratio (%)
Honghu city	Matian village fishery	26	24	92
	Hongcheng fishery	49	46	94
	Wangjialing fishery	19	17	89
	Hongchengyuan fishery	25	23	92
	Xinhe fishery	24	24	100
	Taima lake fishery	28	28	100
	Jinwan fishery	45	43	96
	Fuwan fishery	50	48	96
	Honghu fishery	61	58	95
	Zhangfang fishery	38	36	95
	Hongshi fishery	32	31	97
	Tawau fishery	24	24	100
	Hansha fishery	27	26	96
	Wangling fishery	28	27	96
	Xindi fishery	50	44	88

Jianli city	Chenhu fishery	36	34	94
	Nanhu fishery	25	25	100
	Shengli fishery	24	24	100
	Yayi fishery	16	15	93
	Ya'er fishery	12	12	100

Data resource: Processed from survey.

**Table 4:** Basic characteristics of surveyed samples.

Statistical indicator	Classification indicator	Frequency	Rate (%)
Gender	Male	504	82.8
	Female	105	17.2

Age/years old	40 years old and below	88	14.4
	41–50 years old	127	20.9
	51–60 years old	184	30.2
	60 years old and above	210	34.5

Educational level	Illiterate	79	13
	Primary school	259	42.5
	Junior school	163	26.8
	High school or technical secondary school	72	11.8
	Junior college and above	36	5.9

Family population	Less than 3 people	55	9.1
	3–4 people	184	30.2
	5–6 people	253	41.5
	6 people and above	117	19.2

Fishermen's fishing income	Less than 20,000 yuan	166	27.3
	20,000–50,000 yuan	101	16.6
	50,000–80,000 yuan	100	16.4
	80,000 yuan or more	242	39.7

Cultivated area	Less than 5 acres	354	58.1
	5–15 acres	159	26.1
	16–30 acres	56	9.2
	More than 30 acres	40	6.6

Housing area	Less than 100 m^2^	134	22
	100–200 m^2^	180	29.6
	201–300 m^2^	224	36.7
	300 m^2^ or more	71	11.7

Number of years engaged in fishing (years)	10 years and below	68	11.2
	11–20	117	19.2
	21–30	154	25.3
	31–40	145	23.8
	41–50	78	12.8
	More than 50	47	7.7

Data resource: Processed from survey.

**Table 5:** Exploratory factors of the latent variables.

Variable	AVE
Social capital	0.603
Human capital	0.601
Financial capital	0.519
Physical capital	0.568
Natural capital	0.548

Data resource: processed from survey.

**Table 6:** Test of overall fitness of model.

The fitness of the whole model	*Index of fitting degree*					
	*Absolute fitting value*		*Relative fitting value*			
	CMIN/DF	GFI	RMSEA	NFI	CFI	IFI
Measured value	1.839	0.953	0.062	0.953	0.909	0.919
Ideal value	<5	>0.9	<0.08	>0.9	>0.9	>0.9
Compliance	Compliant	Compliant	Compliant	Compliant	Compliant	Compliant

Data resource: Processed from survey.

**Table 7:** Evaluation index of the model and the result of path test.

Hypothesis	Relationship between latent variables	Path coefficient	*P* value	Direction of influence	Results
H1	Natural capital ⟶ Fishermen's willingness to quit fishing	0.581	0.019	−	Accepted
H2	Physical capital ⟶ Fishermen's willingness to quit fishing	0.498	0.014	−	Accepted
H3	Financial capital ⟶ Fishermen's willingness to quit fishing	0.362	0.024	+	Accepted
H4	Human capital ⟶ Fishermen's willingness to quit fishing	0.592	0.000	+	Accepted
H5	Social capital ⟶ Fishermen's willingness to quit fishing	0.410	0.003	+	Accepted

Data resource: Processed from survey.

**Table 8:** Results of logistic regression model.

*X*	*β*	S.E	Wald	df	Sig.	Exp (*β*)
Social capital (*X*1)	1.395	0.385	8.624	1	0.000	3.549
Human capital (*X*2)	−0.663	0.384	4.542	1	0.026	3.016
Financial capital (*X*3)	−1.251	0.324	7.691	1	0.001	0.403
Physical capital (*X*4)	1.216	0.567	7.954	1	0.004	3.694
Natural capital (*X*5)	0.841	0.268	6.519	1	0.005	0.249
*C*	−3.102	1.381	3.335	1	0.065	0.046

Data resource: Processed from survey.

**Table 9:** Comparative analysis with other research results.

Research team	Time	Study area	Sample size	Estimation method	Estimation results
Lei et al. [29]	2018	Poyang lake	214	Entropy method	1.6966
Pang and Jin [27]	2019	Poyang lake	328	Conditional valuation method	2.58 × 104/a
This research	2022	Honghu lake	609	Willingness survey	66.7%

## Data Availability

The interview data used to support the findings of this study are available from the corresponding author upon request.
